# A Mechanics Study on the Self-Righting of Abalone from the Substrate

**DOI:** 10.1155/2020/8825451

**Published:** 2020-12-10

**Authors:** Yun Zhang, Shanpeng Li, Pingcheng Zuo, Jing Li, Jianlin Liu

**Affiliations:** ^1^College of Pipeline and Civil Engineering, China University of Petroleum (East China), Qingdao 266580, China; ^2^College of Mechanical and Electrical Engineering, China University of Petroleum (East China), Qingdao 266580, China

## Abstract

In this study, we aim to probe the self-righting behavior of abalone on a substrate based on experiments and mechanistic analyses. A successful self-righting process of abalone is observed, and its critical condition in theory can be given in terms of the rotation angle. Then, according to the moment balance and potential energy minimization, the required tension force of the abalone foot for self-righting is derived with respect to the rotation angle. The experimental result also shows that in many cases the abalone cannot finish this self-righting process. Then, measurements on the tolerant strength of abalone muscle and tolerant adhesion strength of the foot on substrate are both conducted. It is judged that the abalone muscle is strong enough, which can provide enough tension force, and thus, the self-righting mainly depends on the adhesion area of the foot on substrate. These findings cast new light on engineering new types of biomaterials and devices, such as marine equipment and soft robotics.

## 1. Introduction

Over millions of years' evolution, many living creatures on earth have developed ingenious structures and functions to adapt to severe wild environments. One magic phenomenon is that a number of organisms have mastered the exquisite skill of attachment or adhesion, which has been studied by many scholars and engineers. For instance, marine creatures such as mussels [1] and barnacles [2, 3] can tightly adhere to the surfaces of ships, rocks, and iron platforms. These two animals can attach on the substrate permanently, as the mucus secreted from their mucous glands acts as a kind of biological viscose. Besides mussels and barnacles, there are many animals in nature that possess the capacity of temporary adhesion, and one typical example is leech. It was reported that the adhesive force of leech generating from the suckers at two ends of its body is bigger than 118 times of its weight, which is really a huge value [4]. Similarly, octopus and clingfish both use suckers depending on atmospheric pressure to create firm attachment [5, 6]. Another typical animal relying on adhesion is gecko, who can run and even jump on the wall to hunt mosquitoes. The adhesion of gecko mainly benefits from the van der Waals force between its feet and the contact surface, as there are numerous seta-based nanofibres distributed on the feet [7–10].

Similar to gecko, the abalone pedal is also equipped with multiscale structures. It has been declared that an adult abalone could produce very high adhesion strength (around 1.2 times the atmospheric pressure) due to setae on the pedal surface, which enable this creature to adhere and crawl on diverse substrates [11, 12]. Obviously, the adhesion ability of abalone can be also governed by the properties of the substrate surface, e.g., wettability, morphology, and material parameter [13]. It should be mentioned that, as the only organ of abalone that directly interacts with the habitat, the pedal is not as tender as it looks; and conversely, it is robust and flexible enough to touch sharp and pointed elements on rock or coral surfaces. Actually when faced with these dangerous surfaces, abalone could nip the sharp or pointed corners without injury, and this posture is beneficial to reduce more than 90% of the stress on its foot [14].

Adhesion can not only assist abalone to crawl on rough surfaces [11, 14] but also make it turn over to avoid the dangers of predators. Actually, the overturned posture is fateful for most animals, as this dangerous behavior could cause their asphyxia and even death. And therefore, in order to avoid invading, these animals can regain upright postures immediately when they are flipped, which is called self-righting. It can be seen that many terrestrial and aquatic organisms, such as turtles, insect, sea star, and locust, tend to accomplish the self-righting process by means of a rolling motion using their legs and heads [15–19]. Normally, abalone in oceans adheres on such surfaces as ship, rock, and marine construction with a supine posture [20]. However, once the abalone is faced with threats, even though it attaches very quickly on the surface, it could occasionally be peeled off from the substrate. Even though the animal clings tightly on the substrate, its supine posture makes the inversion possible once abalone falls from the adhesion surface. When the abalone lands with flipped posture, it is vulnerable to predators, and it must try to turn over to protect itself.

There are not too few studies on the self-righting behavior of abalone which have been made up to now. The self-righting behavior of the abalone is also significant for the aquaculture. The related work is as follows. Ahmed et al. pointed out that, during the abalone culture, the performance in self-righting of abalone juveniles plays a very important role in the survival rate, as failed righting would result in exhaustion or being killed [21]. Braid et al. have recommended using the self-righting time of abalone on substrate as one parameter to estimate the healthy condition of abalone [22]. It was also found that abalone prefers solid surfaces rather than loose ones, such as the sand-like substrate, as the firm attachment on solid is one key factor to realize self-righting [14, 21]. Although some efforts have been made on the abalone self-righting studies, quantitative investigations based on mechanics have not been reported as yet. Consequently, the current exploration is directed towards a comprehensive survey on how the abalone overcomes the bottleneck in the self-righting process, in the light of force analysis and energy calculation.

The outline of this article is organized as follows. In Section 2, a successful self-righting process of abalone was observed, and the geometric configuration during rotation was characterized. In Section 3, the critical geometry condition in theory was given, and then, the required tension force during pulling was calculated by the moment balance and energy minimization. In Section 4, the tolerant strength of the abalone muscle and tolerant adhesion strength of the pedal on substrate were both measured, which were compared with the required tension force. Finally, conclusions were made based on the experiment and mechanistic analysis.

## 2. Materials and Methods

### 2.1. Abalone Self-Righting

The abalone *Haliotis discus hannai* used in the experiment exists widely in the Chinese coasts along the Bohai Bay and Yellow Sea. All the abalones in the experiment were artificially cultured edible, which were bought from a marine aquaculture plant located in the coastal region in Qingdao of China. All alive specimens (15 abalones) are 2~4 years old, where the longitudinal length of the shell is 5~7 cm and the mass ranges from *M* = 25 g to 70 g. To keep the seawater clean and cool (19~20°C), the abalones were fed in a 480 L tank which is equipped with a thermostat to form a filtering and water circulating system. The seawater is made of fresh water and sea salt (Guangzhou Yier Animal Automation Equipment Co. Ltd.). Two types of armored glass with different sizes were utilized as substrates. The dimensions of the rectangular glass are 76.2 × 25.4 × 1 mm^3^ and 200 × 200 × 8 mm^3^, respectively. Moreover, sands collected on the beach of Tangdao Bay in Qingdao were used as the second type of substrate, which was put into a box with a flat bottom surface. After being washed and sterilized by concentrated alcohol and fresh water, all of the substrates on which abalones were raised were placed in cages made of fishing net and were sunk at the bottom of the tank. To make sure that each abalone could adapt to the new environment, all individuals were held on these cages for seven days at least. The abalone was fed with kelp every other three days before the experiment, to ensure that all abalones are healthy [14, 23–25].

To observe the self-righting of the abalone, the animal was first flipped on the substrate, as shown in Figure 1. A camera (Nikon D720, 4000 × 6000 dpi) was used to record the whole motion of the abalone. Another camera (FUJIFILM X-E2) was utilized to record the adhesion area from the bottom view, and the value of the contact area could be measure by the free software ImageJ. All the self-righting experiments were conducted in stagnant water, and the influence of fluid flow was ignored. The experiment was performed under room temperature.

### 2.2. Mass Center Measurement

The mass center was measured according to the suspension method in elementary mechanics. First, the abalone mass was measured by an electronic scale (YP2002, Shanghai Scientific Instruments Co. Ltd.). Then, the animal was immersed in 5% MgCl_2_ in seawater [26, 27]. After that, its viscus was taken out of the abalone shell and weighted by the electronic scale. The volume was measured by means of the drainage approach, and the density can thus be obtained. The area of the viscus was measured by an anticorrosive film tightly covered on the viscus, as the air between them was expelled. Then, we cut the film along the viscus boundary, next we took photos by the camera, and finally we measured the area in use of the free software ImageJ. The length of the abalone shell was measured by a thin cord around the contour of the shell, and then, the length of the shell could be measured by a ruler. To conduct the suspension experiment, a soft cord was used, and one end of it was glued on the edge of the abalone shell by super glue (HJ-403 from Dongguan Gu Bang Adhesive Co. Ltd.). The other end of the cord was fixed on the iron support stand. The extended lines of the cord for the first and second time of suspension experiment would intersect at one point, which is just the position of mass center.

### 2.3. Tolerant Strength Measurement

The tolerant strength of the abalone muscle and tolerant adhesion strength between the foot and substrate were both measured by the universal testing machine (UTM-1432, Cheng De Jin Jian Testing Instrument Co. Ltd.).

Firstly, we measured the tolerant strength of the abalone muscle itself. We cut 5 rectangular samples from the sole foot of anaesthetized abalones (25.29 g, 25.45 g, and 25.56 g), with the dimension of 35 × 9 × 3 mm^3^. The two ends of the sample were clamped by the fixture in the universal testing machine (UTM-1432). The loading velocity was kept 20 mm/min, and the tolerant adhesion strength can be obtained as [*σ*_1_] = 18.07 × 10^4^ ± 32433 Pa (Figure 2(a)).

Next, we measured the tolerant adhesion strength of the abalone foot on substrate. The armored glass of 200 × 200 × 8 mm^3^ on which the whole abalone foot adheres was fixed on the sample platform of the universal testing machine. The whole foot of the abalone can be divided into three parts, i.e., the front, middle, and rear parts. As it was observed that the rear part of the foot plays the main role during the self-righting process, we then measured the adhesion strength of the rear part. If a stimulation is exerted on the abalone, it clings tightly onto the surface by using the rear foot. The camera was utilized to record the adhesion state, and the adhesive area can be figured out by the software ImageJ. Then, the self-developed three-pronged steel jaw clamped by the upper fixture of the machine was adopted to hold the abalone shell, as shown in Figure 2(b). The tension force was applied to pull the abalone from the substrate, with the velocity of 20 mm/min, and the tension process can be viewed as in a quasistatic state [28, 29]. The adhesion strength of the rear part of the abalone foot (taken from the abalone of 25.29 g) can thus be measured, and the experiment was performed 10 times altogether. To make the abalone have an adequate rest, each test was conducted every 60 minutes. The average tolerant adhesion strength of the rear part of the abalone foot is given as [*σ*_2_] = 0.021 ± 0.0076 MPa. We also measured the total adhesion strength of the whole foot with the value of 0.0276 ± 0.0089 MPa. Evidently, these two kinds of adhesive strengths are of very close values, and maybe this is the reason that the abalone mainly uses its rear part of the foot to adhere on the surface. As a comparison, we also measured the adhesion strength of abalone on sands in use of the same equipment, and the result shows that the adhesion strength of the abalone is zero in this case.

## 3. Results

### 3.1. Critical Angle

The whole self-righting of abalone is shown in Figure 1, where it can be divided into three stages. Without loss of generality and for the convenience of modeling, a two-dimensional (2D) model is established to disclose the mechanism. When the abalone is flipped on the substrate, it will feel uncomfortable and tends to return its body instantly. Consequently, the animal begins to extend its whole pedal to seek a suitable place for adhesion (Figure 1(a)). The experiment shows that the strain of the pedal can reach 0.65 ± 0.13, which is even bigger than that of pufferfish stomach (with the value of 0.5) [28]. This large deformation ensures the pedal to adhere to a very wide area around its body. Once the target place is found, the abalone pedal can adhere on it with a small area of the rear portion. After that, the abalone starts to pull its body by using its foot, where its shell begins to rotate on the substrate. The rotation angle *α* is defined as the angle between the A–A′ line and the horizontal surface. It can be seen that initially one point on the profile of the shell contacts the substrate, and when the rotation angle attains to a transition angle *α*_0_, the shell contacts the surface with the fulcrum point A′. Thus, the first stage for the turnover of the abalone is in the range of 0 < *α* < *α*_0_ (Figures 1(a) and 1(b)). The rotation angle corresponding to the state when the line CA′ is vertical to the surface is defined as *α*_*c*_, and in geometry, this is the critical state for abalone self-righting. Thus, when *α*_*c*_ > *α* ≥ *α*_0_, it is considered as the second stage (Figures 1(b) and 1(c)). In the third stage, i.e., when 180° > *α* ≥ *α*_*c*_, the gravity effect can provide the driving force for motion, and the animal can automatically accomplish the remaining rotation, as shown in Figure 1(d).

The question left is to determine the value of *α*_*c*_, and we take an abalone with the mass 25.29 g to analyze. Without loss of generality, the profile of the A–A′ cross section is abstracted as an ellipse, with the long axis 2*a* and short axis 2*b*, and this 2D model is shown in Figure 3.

Refer to the Cartesian coordinate system *o*‐*xy*, where the origin *o* is located at the lowest point of the shell profile when line A–A′ is horizontal. The function of the shell profile is expressed as

(1) $$\begin{array}{c} y=b-b\times \sqrt{1-\frac{x^{2}}{a^{2}}}. \end{array}$$

The coordinate of the mass center C could be thus calculated as

(2) $$\begin{array}{c} y_{\text{C}}=\frac{\int_{A}\rho_{v}ydA+\int_{l_{1}}\rho_{s}yds}{\rho_{v}A+\rho_{s}l_{1}}, \end{array}$$

where *A* and *l*_1_ are the area and arc length of the system consisting of the shell and viscus. The parameters *ρ*_*v*_ and *ρ*_*s*_ are the surface density of the viscus and linear density of the shell, which are measured as 1.377 g/cm^2^ and 2.697 g/cm, respectively. Therefore, the value of *y*_C_ could be calculated as 0.0038 m. It is very close to the result measured by the suspension experiment, which is 0.004 m. During the righting procedure (Figure 3), it is obvious that *α*_*c*_ could be gained by *α*_*c*_ = ∠CA′E + 90°, with the value of 102.68°.

### 3.2. Required Tension Force in Self-Righting

For a successful self-righting process of abalone, the required tension force of the foot can be derived in theory. Although in the first stage (0 < *α* ≤ *α*_0_) and the second stage (*α*_0_ < *α* ≤ *α*_*c*_) (Figure 1) the shell contacts the surface at different points, the moment balance can lead to the same equation, which reads

(3) $$\begin{array}{c} T=\left(Mg-F_{b}\right)\frac{l_{2}l_{4}}{{hl}_{3}}, \end{array}$$

where *g* is the gravitational acceleration, *F*_*b*_ is the buoyancy, *l*_2_ is the force arm of the gravity, *l*_3_ is the length of line A′B, *l*_4_ is the length of the abalone foot represented by the segment EB, and *h* is the distance between point E and the substrate. These parameters can be, respectively, written as

(4) $$\begin{array}{c} l_{2}=\left\{\begin{array}{cc} \frac{a^{2}b}{\sqrt{a^{4}+x^{2}\left(b^{2}-a^{2}\right)}}+\frac{y_{c}}{a}\sqrt{\frac{a^{2}-x^{2}}{a^{4}+x^{2}\left(b^{2}-a^{2}\right)},} & \left(0<\alpha \leq \alpha_{0}\right),\\ \sqrt{\frac{l^{2}}{4}+{\left(h_{0}-y_{c}\right)}^{2}}\cos\left(\alpha -\theta \right), & \left(\alpha_{0}<\alpha <\alpha_{c}\right), \end{array}\right. \end{array}$$

(5) $$\begin{array}{c} l_{3}=\left\{\begin{array}{cc} \frac{xl-2x}{a}\sqrt{a^{4}-4b^{4}}, & \left(0<\alpha \leq \alpha_{0}\right),\\ \text{Constant}, & \left(\alpha_{0}<\alpha <\alpha_{c}\right), \end{array}\right. \end{array}$$

(6) $$\begin{array}{c} l_{4}=\left\{\begin{array}{cc} \sqrt{{\left(l_{3}-\frac{h_{0}-y}{\sin\alpha }+\frac{h}{\tan\alpha }\right)}^{2}+h^{2}}, & \left(0<\alpha \leq \alpha_{0}\right),\\ \frac{1}{2}\sqrt{{\left(l\cos\alpha +l_{3}\right)}^{2}+{\left(l\sin\alpha \right)}^{2}}, & \left(\alpha_{0}<\alpha <\alpha_{c}\right), \end{array}\right. \end{array}$$

(7) $$\begin{array}{c} h=\left\{\begin{array}{cc} a\left(b-h_{0}-\frac{ab}{\sqrt{a^{2}-x^{2}}}\right)\sqrt{\frac{a^{2}-x^{2}}{a^{4}+x^{2}\left(b^{2}-a^{2}\right)}}, & \left(0<\alpha \leq \alpha_{0}\right),\\ \frac{l\sin\alpha }{2}, & \left(\alpha_{0}<\alpha <\alpha_{c}\right), \end{array}\right. \end{array}$$

where *h*_0_ is the length of the segment *o*E, *l* is the length of the segment AA′, and the angle *θ* = 12.68° according to the geometric calculation. For comparison, the required force in theory can also be deduced in the light of energy approach. According to our measurements, the self-righting angular alteration rates of these three stages are 13.5 ± 0.7°/s, 12 ± 1.03°/s, and 90 ± 1.3°/s, respectively. Therefore, in the first and second stages, the kinetic energy is just on the order of 10^–11^ J, and that of the potential energy due to gravity is on the order of 10^–4^ J; obviously, the dynamic effect can be ignored. The potential energy of the abalone due to gravity reads

(8) $$\begin{array}{c} E={Gh}_{1}\left(\alpha \right), \end{array}$$

where *h*_1_ is the vertical height between the mass center C and the substrate (Figure 3), which is expressed as

(9) $$\begin{array}{c} h_{1}=\left\{\begin{array}{cc} a\left(b-y_{\text{C}}-\frac{ab}{\sqrt{a^{2}-x^{2}}}\right)\sqrt{\frac{a^{2}-x^{2}}{a^{4}+x^{2}\left(b^{2}-a^{2}\right)}}, & \left(0<\alpha \leq \alpha_{0}\right),\\ \sqrt{\frac{l^{2}}{4}+{\left(h_{0}-y_{\text{C}}\right)}^{2}}\sin\left(\alpha -\theta \right), & \left(\alpha_{0}<\alpha <\alpha_{c}\right). \end{array}\right. \end{array}$$

It should be mentioned that the whole energy of the system also includes the elastic energy, which has been ignored as the elasticity of abalone foot has not been considered. Then, the tension force can be obtained from the derivative of the potential energy:

(10) $$\begin{array}{c} T=-\frac{dE}{{dl}_{4}}. \end{array}$$

The variations of the tension force and potential energy with respect to the rotation angle are depicted (Figure 4). It shows that the two tension force curves based on the moment balance and energy principle are very close, which indicates that they are consistent. It can be seen that, at the state with transition angle, the tension force has the maximum value, corresponding to the inflection point on the energy curve. Although the force curve is not smooth, it is continuous.

In the first stage, the tension force increases with the increase of the rotation angle, and in the second stage, it decreases with the rotation angle. In the first stage, the tangential line of the force curve becomes bigger with the increase of the rotation angle, and it arrives at the maximum value at the transition angle. In the second stage, the tension force decreases very quickly and becomes zero when the rotation angle is equal to the critical angle. At this critical point, the potential energy reaches the peak, as the mass center gets the highest position. The tension force disappears at this point which implies that beyond this critical angle, there is no need to apply driving force on the abalone.

It is also noted that there are some discrepancies between these two results in Figure 4, and the reason should naturally lie in the expression of the whole energy. In particular, the elastic energy in the first stage is minute as the tension of abalone foot is not obvious, and in the second stage, this effect works significantly and causes discrepancies. However, the moment balance analysis which is accurate has the close result with that of the energy method. This indicates that while the simplification of energy terms leads to the discrepancy, this treatment can be acceptable.

## 4. Discussion

The previous analyses lay a very thorough landscape for the abalone self-righting, and the critical condition is clearly dictated by geometry conditions. However, we observe that most of the self-righting processes of abalone could be realized in the experiment, and in many cases, the animal could not reach the critical state *α* = *α*_*c*_. The maximum angle in these failure processes for self-righting is defined as *α*_*f*_, which is smaller than *α*_*c*_. The statistical results of *α*_*f*_ with respect to different mass *M* are counted (Figure 5) and those of the transition angle *α*_0_ are also given. It is noted that the transition angle *α*_0_ is nearly a constant, with the value of 53.94 ± 2.63°, which implies that this angle is independent of the body size.

This phenomenon makes us further consider the strength of the abalone pedal, i.e., if the abalone has enough capability to produce tension force. The first problem is that the tension force *T* must be compared with the tolerant force *F*_1_ that the abalone muscle can provide. If *F*_1_ < *T*, the muscle is not strong enough, and it will break under the action of this load; thus, it cannot realize the self-righting. The tolerant force is given as

(11) $$\begin{array}{c} F_{1}=\left[\sigma_{1}\right]S_{1}, \end{array}$$

where [*σ*_1_] = 18.07 × 10^4^ ± 32433 Pa is the tolerant strength of the muscle and *S*_1_ is the cross-sectional area of the adhered pedal. As a result, the tolerant force *F*_1_ can be calculated as 4.88 N, which is much bigger than *T*_max_ = 0.085 N (Figure 4). The strength check shows that the abalone muscle is strong enough, and it is impossible to break during the self-righting process. Therefore, the failure reason for self-righting must be due to the strength of the adhesion spot.

Indeed, the attachment force of the foot on substrate is expressed as

(12) $$\begin{array}{c} F_{2}=\left[\sigma_{2}\right]S_{2}, \end{array}$$

where *S*_2_ is the adhesion area of the foot. The adhesion strength of abalone [*σ*_2_] = 0.021 ± 0.0076 MPa has been proved a constant on a particular continuum substrate, such as glass and steel [13]. As a result, the variation of the adhesion area directly affects the adhesion force, which can govern the self-righting result.

Our experiment also shows that, once the substrate cannot offer sufficient adhesion area, e.g., sand, the self-righting is doomed to failure. Altogether, the geometric condition is just the goal for a successful self-righting in a perfect case, but it needs the mechanics condition to support this goal. That is to say, only when the geometric condition and mechanics condition are both satisfied can the self-righting procedure be realized successfully. For example, three experiments on the adhesion area of the abalone (*M* = 25.29 g) with respect to the rotation angle were presented (Figure 6), and the theoretical curve for a successful self-righting as a critical state was compared. It can be seen that, in the two experiments on the failed self-righting, the adhesion area curves are crossed with the critical curve in theory; thus, in these two cases, the maximum rotation angle can only attain *α*_*f*_ = 24° and 55°, which are smaller than *α*_*c*_. During this situation, the adhesion areas of abalone foot are *S*_2_ = 0.23 mm^2^ when *α*_*f*_ = 24° and *S*_2_ = 3.46 mm^2^ when *α*_*f*_ = 55°; and the corresponding adhesion forces are *F*_2_ = 0.0048 N and *F*_2_ = 0.073 N, respectively, which are smaller than the maximum value of the required tension force *T*_max_ = 0.085 N (Figure 4). Therefore, due to the healthy reason or response to ambient environments, the abalone can only make a very small adhesion area at spot, which normally leads to the failure of self-righting. On the contrary, a successful self-righting of abalone is also displayed (Figure 6). In this case, the adhesion area *S*_2_ is much bigger than the theoretical one, and the adhesion force *F*_2_ is calculated as 3.29 N, which is much bigger than *T*_max_ = 0.085 N (Figure 4). It was verified by the experiment that in this case the adhesion area *S*_2_ amounts to a big value at the beginning of the righting, which guarantees that the abalone can generate sufficient adhesion force to pull itself up to *α*_*c*_.

## 5. Conclusion

In conclusion, we have performed a comprehensive study on the self-righting of abalone on the substrate. First, the whole self-righting snapshots were observed by a camera, and the critical geometric condition in theory was given in terms of the rotation angle. Then, according to the moment balance and potential energy minimization, the required tension force of the abalone foot in theory was derived with respect to the rotation angle. The experimental result also shows that in many cases the abalone cannot finish this self-righting process due to some physiological reasons. The measurements on the tolerant strength of muscle and tolerant adhesion strength of the foot on substrate were both performed to explore the failure reason. It is found that the abalone muscle is strong enough and can provide sufficient tension force, and as a consequence, the self-righting mainly depends on the adhesion area of the foot on substrate.

It is expected that this self-righting mechanism can be generalized to analyze the similar behaviors of many creatures, such as turtle, beetle, and cicada. The mechanics model can also provide some inspirations on the design of mechanical structures for machines to stabilize. The constitutive relationship of the abalone foot is beneficial to engineering new bionic devices. The motion of the abalone can be extended to design robotics, and its complex trajectory can be referred to. To enrich the study, some other parameters, such as smoothness, wetting property of the substrate, and dynamic effect, can be taken into consideration in the future. The constitutive relationship of the foot will not be limited to the linear Hookean material, and the viscoelastic properties should also be considered.

## Figures and Tables

**Figure 1:** Snapshots and schematics of a successful abalone self-righting process, which are divided into three stages.

**Figure 2:** Strength measurement experiment on one abalone (*M* = 25.29 g). (a) Experimental setup and result of the tolerant strength of the abalone foot muscle. (b) Experimental setup and result of the adhesion strength of the abalone foot on substrate.

**Figure 3:** Two-dimensional model of the self-righting process, where point C is the mass center, B is the adhesion point, and A′ is the fulcrum point at the transition state.

**Figure 4:** Dependence relationships between the required tension force and potential energy and the rotation angle *α* in the whole self-righting process. Line 1 is the tension force derived by the moment balance, and line 2 is that from the potential energy minimization. Line 3 is the potential energy curve due to gravity.

**Figure 5:** Measurement results of the maximum failure rotation angle *α*_*f*_ during the self-righting process and the transition angle *α*_0_ with the average value of 53.94°.

**Figure 6:** Three examples in the self-righting process, where the line with rectangular points is a successful process and the lines with triangular and circular points are failed processes. The solid line represents the critical curve to distinguish these two behaviors.

## Data Availability

All data included in this study are available upon request by contact with the corresponding author.
